The article "Study of Complexity Systems in Public Health for Evaluating the Correlation between Mental Health and Age-Related Demographic Characteristics: A General Health Study" was published in 2022. Journal: J Healthc Eng.

# Study of Complexity Systems in Public Health for Evaluating the Correlation between Mental Health and Age-Related Demographic Characteristics: A General Health Study

**DOI:** 10.1155/2022/2117031

**Published:** 2022-04-06

**Authors:** Fereshte Haghi, Shadi Goli, Rana Rezaei, Fatemeh Akhormi, Fatemeh Eskandari, Zeinab Nasr Isfahani

**Affiliations:** ^1^Shahid Beheshti OB&GYN Hospital Isfahan University of Medical Sciences, Isfahan, Iran; ^2^Nursing and Midwifery Sciences Development Research Center, Najafabad Branch, Islamic Azad University, Najafabad, Iran; ^3^Department of Midwifery, Shoushtar Faculty of Medical Sciences, Shoushtar, Iran; ^4^Department of Midwifery, Ahvaz Jundishapur University of Medical Sciences, Ahvaz, Iran

## Abstract

The main objective of this study is to evaluate the quality of nurses' work lives and mental health during outbreaks. We also use the General Health Questionnaire–28 and Walton's QWL technique to assess the association between these two and their dimensions with demographic variables and each other. First, 165 nurses from COVID-19 medical centers in Iran filled surveys for this research. In an SPSS program, the data were examined. There was a strong link between mental health and age-related demographic factors. There was no evidence of a link between the quality of nurses' work life and their psychological health. However, there was a strong link between somatic symptoms and fair and appropriate compensation, as well as constitutionalism. The worst situations for work life quality were linked to the whole living area dimension. In contrast, the worst conditions for mental health were linked to the somatic symptoms dimension.

## 1. Introduction

In December 2019, an acute respiratory syndrome caused by SARS-CoV-2 caused a global pandemic in Wuhan, China, where almost the entire human community has been directly affected by the disease or associated safety social restrictions. Numerous studies have been published on the mechanism of action of this coronavirus and its individual and social effects and consequences, which indicate the occurrence of physical disease in the form of clinical complications and manifestations such as fever, chills, sore throat, contusion, cough, respiratory problems, vomiting, and diarrhea [1], as well as psychological complications such as fear and anxiety [2]. Of course, clinical complications have affected patients, and psychological complications have affected both patients and nonpatients. The pandemic has had a tremendous impact on various occupations. It has imposed different consequences on the working community, active in various business sectors [3]. COVID-19 has attracted special international attention as a serious threat to global public health. The increasing prevalence of this disease and the prolongation of the disease process have made the activities of the medical staff exhaustive [4]; Thus, with the over-admission of patients in medical centers, the availability and readiness of the medical staff is a determining factor in overcoming the crisis [5]. Considering that various studies and reports indicate the effect of health care providers' satisfaction on patient satisfaction [6–11] and on the other hand, job satisfaction has a two-way relationship with the mental and psychological condition of employees [12], it is essential to consider psychological conditions and their improvement methods in the medical center.

The article "Study of Complexity Systems in Public Health for Evaluating the Correlation between Mental Health and Age-Related Demographic Characteristics: A General Health Study" was published in 2022. Journal: J Healthc Eng.

According to the World Health Organization definition, mental health is “a state of wellbeing in which the individual realizes his or her abilities, can cope with the normal stresses of life, can work productively and fruitfully, and can make a contribution to his or her community.” Good mental health is one of the pillars of health and is necessary for a useful, effective, and satisfying life [13]. Quality of work life (QWL) is essential for attracting and retaining employees. When an organization provides a good QWL for employees, it intends to retain employees [14]. Quality of work life is one issue that affects almost all people regardless of the situation. In hospitals and medical centers, the quality of hospital services will not be guaranteed without the participation of nurses [15]. Various factors such as incompatibility and dissatisfaction with work, stress, fatigue, illness, and lack of leisure time of nurses affect their behavior [16]. Nurses who have dealt with patients for a more extended period are more likely to be vulnerable. Critical and painful patients, dying patients, complex equipment, inappropriate behaviors of patient companions, patients' reactions, and many other issues give different aspects to nurses' work, and such conditions affect burnout, job satisfaction, and the tendency of nurses to continue working [17]. These characteristics in the workplace increase stress and the risk of mental disorders [18]. Nursing is one of the 130 most stressful occupations and is ranked 27th among 130 occupations with a high prevalence of mental disorders [19]. Nurses face several stressful sources such as time, long-term work, change of work shift, insomnia, death observation, malignancy, high patient expectations of nurses, and a low tolerance for error [20]. Job stress can lead to disorders that put nurses at serious risk of mental disorders [21].

From December 2019 onward, medical staff, especially nurses, are under severe pressure. Various waves of COVID-19 have swept across many countries, including Iran. In this situation, not only do medical staff rescue infected patients but they also oversee the entire process of combating health events. In addition to the stress of the job itself, they are involved in a conflict between their safety needs and job requirements. They may be exposed to anxiety, depression, insomnia, and other psychological disorders [22]. High-sensitivity patient care imposes significant physical and emotional burdens, exacerbated by increased workload, staff shortages, and equipment shortages. Direct contact with the patient increases the risk of infection [23]. Meanwhile, the measures taken by the government, especially with an emphasis on social distance and restricting communication and travel outside the workplace, are also significant. Therefore, it is impossible to take many common strategies to reduce stress and anxiety, which increases the responsibility of medical centers to take the initiative and create the appropriate conditions to compensate for the shortcomings. Paying attention to the QWL and improving it is one of the approaches used by organizations. However, the QWL includes several aspects, and consequently, a variety of solutions in this area is considerable.

The article "Study of Complexity Systems in Public Health for Evaluating the Correlation between Mental Health and Age-Related Demographic Characteristics: A General Health Study" was published in 2022. Journal: J Healthc Eng.

It is necessary to properly understand the psychological problems of nurses in the context of the COVID-19 pandemic, the relationship between various problems and mental disorders with different aspects of work life, and to create the right mentality to adopt an appropriate solution. These strategies may vary even concerning the nurses' workplace. From this point of view, it is necessary to conduct the necessary research. According to the explanations provided, it can be said that this study seeks to answer the following questions:

- What are the most important problems and inadequacies related to the quality of work life?
- What are the most important problems and mental disorders?
- What is the correlation between the aspects of quality of work life and mental disabilities?

## 2. Literature Review

Numerous studies have been conducted on mental health and QWL and their relationship. A significant part of these studies goes back to nurses working in medical centers. Javadi-Pashaki and Darvishpour [24] in their study on stress and coping strategies to predict the general health of nursing staff considered 318 nurses working in health centers of Guilan University of Medical Sciences [24]. The results showed that stress and coping strategies could explain about 2.5% of the variance in public health. However, the results showed that coping strategies are significantly more predictive of public health. Accordingly, attention to coping strategies to predict general health in nurses has been highlighted. Mahmoudi [3] studied the economic effect of COVID-19. This model is enhanced with additional characteristics to assess the economic impact of COVID-19 on the labor market. The findings indicate that the US government might employ a straightforward technique to mitigate the harmful effects of COVID-19.

The article "Study of Complexity Systems in Public Health for Evaluating the Correlation between Mental Health and Age-Related Demographic Characteristics: A General Health Study" was published in 2022. Journal: J Healthc Eng.

Zhang et al. [22] in their study of the mental health status of Chinese healthcare-related infection control specialists during the coronavirus outbreak investigated data from 9,228 cases from 3,776 hospitals across China in the form of an online questionnaire. A 12-item Chinese version of the General Health Questionnaire and a Chinese version of the Psychological Capital Questionnaire suitable for medical personnel were used as tools in this study. By performing univariate and multivariate analysis, it was found that the risk of mental health problems is higher with more self-sufficiency and working in a public hospital. Working in a second-degree rather than a third-degree hospital poses a significantly lower risk. However, fewer psychological problems have been observed in single people than in married ones. In addition, fewer working hours per week, hope, and optimism played a role in reducing risk. Hardiyono [25] in their study on burnout of nurses working in the hospital for the treatment of patients with COVID-19 concluded that burnout is present in nurses who were exposed to a large number of patients with the virus [25]. The high workload, and at the same time, the worry of transmitting the virus to themselves and their family members is one of the most important factors that put them under psychological pressure and lead to burnout. Quchan et al., in their study, compared the mental health of nurses working in COVID-19 referral hospitals and regular hospitals [2]. 60 nurses related to the COVID-19 wards and 62 non-COVID-19 nurses participated in the study. A standard public health questionnaire was provided to them online. There was no statistically significant difference between the two groups. However, both groups had poor mental health, which the researchers said was probably due to the pandemic. Sadeghipoor and Moradisabzevar [26] developed a smart toy car to screen children for autism. The findings indicate that the system has an accuracy rate of 85 percent, a sensitivity of 93 percent, and a specificity of 76 percent. The findings are same for boys and girls, indicating that this approach may be widely used by all youngsters.

Dehkordi et al. [27] conducted a study on the effect of COVID-19 disease on anxiety, quality of work life, and fatigue of health care providers in health centers in southwestern Iran. The statistical population includes 181 people directly related to patients and 261 employees in other wards who had no direct contact with patients with COVID-19 [27]. They concluded that both groups' work life quality had decreased, and fatigue and anxiety caused by COVID-19 had increased. However, there is no statistically significant difference between the fatigue caused by the anxiety of the staff involved with COVID-19 and the personnel of other departments. In terms of QWL, no significant difference was observed in other components except for human resource development. The results also showed a statistically significant relationship between the level of component anxiety with QWL and fatigue. Kelbiso et al. [28] have identified and analyzed the determinants of QWL among nurses working in public health facilities in Hawassa, Ethiopia [28]. In this study, 253 nurses from two hospitals and nine health centers participated. Findings showed that at least 60% of nurses were dissatisfied with their quality of work life. This study showed that independent predictors of QWL among the study population were educational status, monthly income, position, and work environment. Abadi et al. [29] used a unique hybrid salp swarm technique and genetic algorithm to schedule nurses to care for COVID-19 patients. Zhang et al. [30] expected that perceived social distance would positively buffer the effect of anger on trust and that gender would moderate the effect of perceived social distance on trust. According to the findings, female participants, but not male participants, sent more money to their counterparts in the low social distance than in the control condition. Women's optimistic risk assessment and consequently greater trust in others may be triggered by the high certainty, higher individual control, and approach motivation associated with anger, according to the findings of both studies. This is due to women's perception of a smaller social distance. Public transportation networks, mobile operators, and mobile phone applications were taken as the three key sources of mobility data by Hu et al. [31]. Sadeghipour et al. (2016) concentrated on facial recognition with the use of an enhanced SIFT algorithm. The results demonstrate that the suggested method outperforms the SIFT. The suggested approach is evaluated by applying it to the ORL database and then comparing it to existing face identification techniques [32]. In order to assess human mobility, four following ways are typically used: public transit-based flow, societal activity patterns, index-based movement data, and social media-derived movement data. Sharifi et al. [33] studied the impact of artificial intelligence and digital style on the industry and energy following COVID-19. According to Chen et al. [34], a Markov chain position predictions model based on multilevel correction was presented. This approach is also helpful in determining the correlation between the variables in the COVID-19 dataset. Ala et al. [35] studied how the whale optimization algorithm and the NSGA-II can be used to optimize appointment scheduling for healthcare systems based on the quality of fairness service provided. According to Hankir et al. [36]; a study protocol is being developed to study an anti-stigma program and long-term reductions in mental health stigma among medical students. Abbas [37] drew on data on coronavirus infections obtained from the Ministry of Health and National Institute of Health Pakistan to conduct his research. This study evaluation includes data provided by the National Institutes of Health, and responses were from all areas of Pakistan, limiting the generalizability of the findings to empirical evidence.

The article "Study of Complexity Systems in Public Health for Evaluating the Correlation between Mental Health and Age-Related Demographic Characteristics: A General Health Study" was published in 2022. Journal: J Healthc Eng.

## 3. Methodology

In the present study, data collection has been performed based on 250 General Health Questionnaire – 28 (GHQ-28) of Goldberg and Hillier [38] and Walton's QWL questionnaire [39] distributed among nurses of ten hospitals in Iran with surgical, orthopedic, COVID-19, intensive care units, emergency, cardiology, and neurology wards. The validity and reliability of both questionnaires have been repeatedly reviewed and found appropriate for screening the QWL and job-related factors [40, 41].

The GHQ-28 questionnaire is multiple choice and has four dimensions: somatic symptoms, anxiety and insomnia, social dysfunction, and severe depression. Its scoring method is in the form of Likert, which has a number between zero and 3 (never = zero, sometimes = 1, most of the time = 2, and always = 3). Each dimension consists of 7 questions. The maximum score in each dimension is 21, and the person's total score is from zero to 84. A higher score indicates lower health. On the other hand, the Walton's QWL questionnaire has eight dimensions in the following order: fair and adequate payment (questions 1, 2, 3), safe and healthy working environment (questions 4, 5, 6), opportunities for continuous growth, and security (questions 7, 8, 9), constitutionalism (questions 10, 11, 12, 13), social dependence of working life (questions 14, 15, 16), the total living space (questions 17, 18, 19), social integration and cohesion in the organization (questions 20, 21, 22, 23), and development of human capabilities (questions 24, 25, 26, 27). This questionnaire is also based on the Likert scale from very low to very high, 1 to 5. The questionnaire does not have a reverse question.

The article "Study of Complexity Systems in Public Health for Evaluating the Correlation between Mental Health and Age-Related Demographic Characteristics: A General Health Study" was published in 2022. Journal: J Healthc Eng.

## 4. Results

Ultimately, 165 nurses working in different wards provided their answers, which the summarized results and related parameters are shown in Table 1. Based on Table 1, The reliability of GHQ-28 based on Cronbach's alpha coefficient is 0.922. The QWL Questionnaire is 0.933, which is excellent.  Table 2 shows the significance of the difference between mental health and QWL for respondents based on their demographic characteristics. As can be seen in this table, according to the medical department, the difference in the mean QWL at the error level of one percent is significant.

At the 5% error level, the difference in the mean for mental health based on employment status is significant. There is no significant mean difference at the 5% error level in other cases.

Additionally, to examine the relationship between age and work experience with mental health and QWL, the Pearson correlation coefficient was used, the result of which is shown in Table 3. As can be seen, the respondents' mental health has a significant positive correlation with their age and work experience.

The ranking of mental health disorders and disorders related to QWL using the Friedman test indicates that Chi-square statistics to evaluate the significance of the difference in the mean rank for mental health and QWL are 162.6 and 755.6, respectively, with an error probability of less than 0.001. The results of this analysis are presented in Tables 4 and 5.

Pearson correlation was also used to examine the relationship between the dimensions of mental health and the dimensions of QWL. The degree of correlation and their significance are shown in Table 6. Even at the 10% error level, there is no significant correlation between QWL and dimensions of mental health. Also, there is no significant correlation between mental health and dimensions of QWL at the same level of error. At the 1% error level, only the correlation between fair and adequate payment and somatic symptoms is significant. However, at the 10% error level, the correlations between somatic symptoms with constitutionalism, anxiety symptoms, and insomnia with the development of human capabilities and social dysfunction with opportunities for continuous growth and security are significant.

## 5. Discussion

The present study is descriptive correlational in terms of purpose and applied in terms of the type of use. It attempts to understand a specific situation in the real world to apply the findings to provide solutions for development and improvement. Therefore, in terms of purpose, it is considered practical. This research is conducted from a descriptive point of view conducted in the field using the data of distributed questionnaires. On the other hand, because it seeks to understand the correlation relationships based on the opinions and desires of individuals, it is considered correlational. The researcher has no role in the relationship between different factors and only uses questionnaires with validity and reliability. In terms of time, it is a cross-sectional study that refers to the experiences and perceptions of nurses up to a specific period. It is also qualitative in terms of data type.

The article "Study of Complexity Systems in Public Health for Evaluating the Correlation between Mental Health and Age-Related Demographic Characteristics: A General Health Study" was published in 2022. Journal: J Healthc Eng.

Further investigation in this regard by focusing on nurses with associate degrees shows that at the level of five percent error, there is a significant correlation between fair and adequate payment with depressive symptoms, opportunities for continuous growth and security with social dysfunction, and the total living space with somatic symptoms. Another essential point in this study is the significant correlation between age and work experience with the mental health of nurses. Due to the negative mental health index, as the age of nurses increases, their mental health deteriorates. However, the correlation between age and work experience with QWL is not significant. Therefore, older nurses are more likely to be psychologically vulnerable and need more support. These results can be delegated by the type of activity or responsibility, which requires further consideration. Regarding the dimensions of mental health, the worst conditions are related to somatic symptoms, and the best conditions are related to depressive symptoms. Regarding the QWL, the worst conditions are related to the total living space, and the best conditions are related to the development of human capabilities. It has been investigated whether specific pandemic protocols have put more pressure on nurses and resulted in fatigue or boredom of the overall living space and confirmed by Sun et al. [42]. The correlation between fair and adequate payment and constitutionalism in QWL with the dimension of somatic symptoms in mental health is significant, indicating that nurses' fatigue is more pronounced concerning the soft aspects of QWL. Consequently, establishing appropriate performance appraisal systems and performance-based pay and rewards can be considered a vital decision-making option. Other issues such as symptoms of anxiety and insomnia and their significant negative relationship with the development of human capabilities are also debatable. Perhaps, more awareness of the pandemic situation has somehow led to anxiety. In this case, reapplying appropriate safety systems by hospitals and medical centers to build trust and confidence in invulnerability can be a desirable option for decision making. Social dysfunction also significantly correlates with opportunities for continuous growth and security. Perhaps, individuals will show more social dysfunction if they have the opportunity to grow and develop in their jobs and professions.

The article "Study of Complexity Systems in Public Health for Evaluating the Correlation between Mental Health and Age-Related Demographic Characteristics: A General Health Study" was published in 2022. Journal: J Healthc Eng.

## 6. Conclusion

In the present study, nurses' mental health status and QWL during the COVID-19 pandemic were evaluated to a limited extent. As expected, the reliability of both questionnaires was acceptable. The study found that if mental health was considered a criterion, the pandemic affected almost all nurses with different demographic conditions. This did not depend solely on the ostensibly involved departments, such as the emergency or COVID-19. However, the study shows that nurses with associate degrees have significantly less mental health.

This study did not identify a significant relationship between age and QWL, same as [43], which is not consistent with the study of [44], stating that there is a close correlation between age and QWL of nurses. The findings of this study are in good agreement with the findings of Bakhshi et al. [14] that there is no significant difference in the mean QWL in different wards of hospitals and medical centers. On the other hand, as mentioned above, the need to pay attention to constitutionalism in this study is evident. In short, it can be said that in the medical centers under study, mental health and QWL in general and within the relevant dimensions are not in good condition. The relationship between them with demographic characteristics and each other indicates the existence of several potential solutions. It is necessary to evaluate the solutions and select the best ones in an appropriate decision-making approach. Suppose the quality of working life improves according to the specific requirements and protocols of the COVID-19 pandemic, it may be hoped that nurses' mental health will improve.

## Figures and Tables

**Table 1:** Summary of information about the respondents and their status in terms of mental health (MH) and QWL.

			Number	Mean	Std. dev.	Max	Min	Median	Mode	%
Age			165	33	7	54	24	32	25	100.0

Work experience			165	9	7	27	0	8	3	100.0

Ward	Orthopedic	MH	11	20.27	7.73	30.00	11.00	18.00	30.00	6.7
		QWL	11	100.45	16.80	122.00	77.00	99.00	82.00	6.7
	Emergency	MH	14	18.71	8.16	38.00	8.00	18.50	19.00	8.5
		QWL	14	103.43	8.99	119.00	92.00	102.00	93.00	8.5
	Surgical	MH	10	30.00	23.90	63.00	6.00	17.50	54.00	6.1
		QWL	10	106.10	9.00	114.00	83.00	106.50	105.00	6.1
	Cardiology	MH	15	24.27	14.27	52.00	9.00	19.00	9.00	9.1
		QWL	15	107.93	14.78	133.00	72.00	109.00	117.00	9.1
	COVID-19	MH	89	27.44	9.25	71.00	9.00	27.00	31.00	53.9
		QWL	89	91.67	11.13	124.00	68.00	93.00	91.00	53.9
	Intensive care units	MH	15	25.67	15.62	60.00	9.00	22.00	9.00	9.1
		QWL	15	98.27	19.05	121.00	64.00	100.00	118.00	9.1
	Neurology	MH	11	25.36	14.08	57.00	9.00	21.00	9.00	6.7
		QWL	11	104.45	17.60	135.00	78.00	105.00	78.00	6.7

Education	Associate degree	MH	18	31.50	9.37	54.00	18.00	30.00	27.00	10.9
		QWL	18	97.61	10.34	121.00	81.00	97.00	97.00	10.9
	Bachelor's degree	MH	128	25.03	11.67	63.00	6.00	23.50	31.00	77.6
		QWL	128	96.20	14.91	135.00	64.00	96.00	94.00	77.6
	Master's degree	MH	19	25.47	15.66	71.00	7.00	21.00	11.00	11.5
		QWL	19	102.32	11.95	121.00	81.00	101.00	96.00	11.5

Employment status	Conscription	MH	39	21.28	11.65	54.00	6.00	18.00	9.00	23.6
		QWL	39	100.10	13.83	121.00	71.00	101.00	118.00	23.6
	Temp-to-perm	MH	27	29.52	12.55	71.00	11.00	28.00	31.00	16.4
		QWL	27	96.11	13.07	124.00	64.00	96.00	91.00	16.4
	Contractual	MH	34	25.09	8.66	40.00	10.00	25.50	32.00	20.6
		QWL	34	92.65	15.44	121.00	66.00	92.50	92.00	20.6
	Permanent	MH	65	27.31	13.00	63.00	7.00	25.00	30.00	39.4
		QWL	65	97.94	14.01	135.00	70.00	97.00	93.00	39.4

Gender	Male	MH	64	23.75	11.47	57.00	6.00	23.50	9.00	38.8
		QWL	64	98.47	13.89	135.00	70.00	99.50	82.00	38.8
	Female	MH	101	27.08	12.31	71.00	9.00	26.00	16.00	61.2
		QWL	101	96.17	14.45	133.00	64.00	96.00	93.00	61.2

MARSTA	Single	MH	42	24.95	13.24	71.00	9.00	21.50	17.00	25.5
		QWL	42	95.17	13.54	124.00	69.00	96.00	92.00	25.5
	Married	MH	123	26.07	11.68	63.00	6.00	25.00	30.00	74.5
		QWL	123	97.71	14.46	135.00	64.00	97.00	91.00	74.5

The article "Study of Complexity Systems in Public Health for Evaluating the Correlation between Mental Health and Age-Related Demographic Characteristics: A General Health Study" was published in 2022. Journal: J Healthc Eng.

**Table 2:** Significance of mean difference for mental health and QWL based on demographic characteristics.

Demographic classification	Significance of mean difference for mental health	Significance of mean difference for QWL
Ward	0.112	Less than 0.001
Education	0.102	0.215
Employment status	0.026	0.143
Gender	0.084	0.313
MARSTA	0.605	0.319

**Table 3:** Significance of correlation between mental health and QWL with age and work experience.

		Mental health	QWL
Age	Pearson correlation	0.276	0.050
	Significance	0.000	0.527

Work experience	Pearson correlation	0.242	-0.026
	Significance	0.002	0.744

**Table 4:** Significance of mean rank difference for mental health disorders.

Mental health disorder	Mean	Std. dev.	Mean rank	Significant
Somatic symptoms	7.70	4.07	2.96	1
Social dysfunction	7.50	2.85	2.95	2
Anxiety and insomnia	6.99	4.42	2.65	3
Severe depression	3.59	3.95	1.44	4
Chi-square statistics for the significance of the difference in mean rank	162.6			
Probability of error	Less than 0.001			

**Table 5:** Significance of mean rank difference for QWL disorders.

Mental health disorder	Mean	Std. dev.	Mean rank	Significant
The total life space	10.42	2.21	2.92	1
Social dependence of working life	10.53	2.17	3.02	2
Opportunities for continuous growth and security	10.61	2.18	3.04	3
Safe and healthy working environment	10.67	2.32	3.19	4
Fair and adequate payment	10.87	2.14	3.44	5
Social integration and cohesion in the organization	14.20	2.54	6.48	6
Constitutionalism	14.12	2.43	6.56	7
Development of human capabilities	15.65	2.34	7.36	8
Chi-square statistics for the significance of the difference in mean rank	755.64			
Probability of error	Less than 0.001			

The article "Study of Complexity Systems in Public Health for Evaluating the Correlation between Mental Health and Age-Related Demographic Characteristics: A General Health Study" was published in 2022. Journal: J Healthc Eng.

**Table 6:** Degree of correlation and their significance.

		Somatic symptoms	Anxiety and insomnia	Social dysfunction	Severe depression	Total mental health
Total QWL	Pearson correlation	−0.097	0.015	−0.051	0.017	−0.034
	Significant error	0.217	0.844	0.514	0.833	0.669

Fair and adequate payment	Pearson correlation	−0.207^∗^	−0.089	0.034	0.113	−0.057
	Significant error	0.008	0.258	0.668	0.147	0.467

Safe and healthy working environment	Pearson correlation	−0.100	0.025	−0.055	−0.022	−0.045
	Significant error	0.199	0.746	0.485	0.775	0.567

Opportunities for continuous growth and security	Pearson correlation	−0.032	0.067	−0.141	−0.054	−0.037
	Significant error	0.687	0.393	0.070	0.491	0.635

Constitutionalism	Pearson correlation	−0.150	−0.040	−0.027	−0.051	−0.089
	Significant error	0.054	0.608	0.732	0.512	0.257

Social dependence of working life	Pearson correlation	−0.077	−0.049	0.042	0.043	−0.020
	Significant error	0.326	0.529	0.595	0.587	0.797

The total life space	Pearson correlation	−0.044	0.002	−0.094	−0.037	−0.049
	Significant error	0.572	0.985	0.228	0.634	0.533

Social integration and cohesion in the organization	Pearson correlation	−0.091	0.038	−0.079	0.022	−0.028
	Significant error	0.246	0.632	0.314	0.777	0.719

Development of human capabilities	Pearson correlation	0.099	0.133	0.008	0.095	0.115
	Significant error	0.208	0.089	0.915	0.224	0.141

## Data Availability

The data are available and can be provided over the email queries directly to the corresponding author (nasrisfahani.z@ajums.ac.ir).
